# Analysis and Recognition of Clinical Features of Diabetes Based on Convolutional Neural Network

**DOI:** 10.1155/2022/7902786

**Published:** 2022-07-29

**Authors:** Rui Wang, Ping Li, Zhengfei Yang

**Affiliations:** ^1^Institute of Traditional Chinese Medicine, Ningxia Medical University, Yinchuan 750000, China; ^2^Weifang Engineering Vocational University, Weifang, Shandong Province 262500, China

## Abstract

Diabetes mellitus is a common chronic noncommunicable disease, the main manifestation of which is the long-term high blood sugar level in patients due to metabolic disorders. However, due to excessive reliance on the clinical experience of ophthalmologists, our diagnosis takes a long time, and it is prone to missed diagnosis and misdiagnosis. In recent years, with the development of deep learning, its application in the auxiliary diagnosis of diabetic retinopathy has become possible. How to use the powerful feature extraction ability of deep learning algorithm to realize the mining of massive medical data is of great significance. Therefore, under the action of computer-aided technology, this paper processes and analyzes the retinal images of the fundus through traditional image processing and convolutional neural network-related methods, so as to achieve the role of assisting clinical treatment. Based on the admission records of diabetic patients after data analysis and feature processing, this paper uses an improved convolutional neural network algorithm to establish a model for predicting changes in diabetic conditions. The model can assist doctors to judge the patient's treatment effect by using it based on the case records of inpatient diagnosis and treatment and to predict the risk of readmission of inpatients after discharge. It also can help to judge the effectiveness of the treatment plan. The results of the study show that the model proposed in this paper has a lower probability of misjudging patients with poor recovery as good recovery, and the prediction is more accurate.

## 1. Introduction

Diabetes is a common chronic noncommunicable disease. Metabolic disturbances in patients can lead to chronically high blood sugar levels in patients. Since the disease is not easy to cure, the long-term high blood sugar level of the patient has brought serious harm to the patient's kidney, cardiovascular, and nervous system, resulting in many complications, which has brought great harm to the patient's physical and mental health [1, 2]. However, according to the World Health Statistics Report released by the World Health Organization in 2017, about 40 million people died of chronic noncommunicable diseases in 2015. Among them, diabetes is the fourth leading cause of death in humans. According to the report, about 80% of people with diabetes are in low- and middle-income countries. Therefore, it is beneficial for diabetic patients, especially those in low- and middle-income countries, to carry out diabetes prevention and control work and help patients improve treatment efficiency [3, 4].

However, there are many problems in the prevention and treatment of diabetes. The traditional treatment of diabetes is based on the medical experience and medical knowledge of doctors [5, 6]. However, according to statistics, by the end of 2017, the total number of health personnel in China was 11.749 million, including 3.39 million practicing (assistant) doctors and 901,000 rural doctors. Although there are a large number of practitioners, compared with the goals in the “Healthy China 2030” plan proposed by China, the number of doctors is far from enough, and some doctors in areas with limited medical resources have a low level of education, although the number of rural doctors is limited [7, 8]. Therefore, some patients in areas with limited medical resources cannot obtain efficient treatment plans or long-term follow-up treatment. Physicians may not be able to monitor the treatment effect of patients in place and cannot adjust treatment plans in a timely and effective manner, thus delaying the treatment opportunity of some patients. However, physicians hope to improve the efficiency of treatment in various ways, so that more patients can receive better treatment and improve the quality of patients' lives [9, 10]. The treatment effect and condition monitoring of diabetic patients are mainly focused on changes in blood sugar levels. Few studies have focused on predicting treatment outcomes for hospitalized patients; however, information on patients' hospitalizations is crucial for patient recovery.

The incidence of diabetic retinopathy in diabetic patients is relatively high. The patients have no obvious symptoms of discomfort in the early stage, and the patients' vision will be affected in the middle stage of the disease course, and there will be transient blurred vision during this period. It will soon return to normal, but patients are often unusual, so that long-term blurred vision, blood shadows, and floating mosquitoes appear in the later stage, resulting in irreversible vision damage and gradually causing vision loss [11, 12]. If diabetic patients have regular fundus examinations and treatment at the early stage of the disease, it may completely eliminate the risk of blindness. Therefore, early screening of diabetic retinopathy and timely treatment for diabetic patients are very necessary [13, 14]. Therefore, it is of great significance to explore the potential medical laws in medical data to assist doctors in understanding the treatment effect and disease trend of patients.

In recent years, due to the advancement of medical informatization and the development of information technology, it is possible to realize the above-mentioned target of diabetes treatment. Due to the realization and popularization of electronic medical records, patients who go to the hospital will leave detailed records such as diagnostic reports at various stages of their diagnosis and treatment in the electronic medical records, physical examination indicators, and other detailed records [15, 16]. These records hide a large number of rules for the diagnosis and treatment of diabetes. These rules can assist some inexperienced or limited medical practitioners in the diagnosis and treatment work and help doctors to formulate accurate and effective treatment plans for patients. The treatment effect of the disease is tracked [17, 18].

In the past, retinal image processing required many stages, and at each step, retinal image processing required at least one computer vision technique. At the same time, the complexity of retinal samples and the influence of various lesions increase the difficulty of their processing. Force majeure external factors make the processing of retinal images cumbersome and require further judgment based on original medical knowledge. In retinal processing, errors in one process or unsatisfactory results can increase the difficulty of the next step and reduce the accuracy of image classification tests. In developed countries with a high incidence of diabetes, many universities and research institutes have been studying how to conduct diabetic retinopathy (DR) screening. The current research is mainly limited by the following aspects: (1) the quality of fundus retinal images. Since the resolution, contrast, saturation, brightness, and other indicators of the acquired image are easily affected by some conditions such as sunlight, camera, hardware, and the experience of the imaging operator, the image quality of the completed retinal images will be uneven. The current situation is uneven, and the quality of some images is quite different. (2) The grading of retinal images is not very clear, and some small changes may affect the judgment of grading, which makes it difficult to label the image grading. (3) The structure of the fundus retina is complex, and the use of traditional machine learning algorithms has high requirements for feature extraction, and information extraction is difficult. All in all, the researchers have achieved good empirical results by examining the existing diabetes data.

Retinal pathological images play an important role in medical diagnosis. Doctors can use this to determine the stage of the disease, and accurate classification of retinal images plays an important role in the treatment of DR. Therefore, researchers at home and abroad have devoted themselves to the research of DR classification with great enthusiasm and developed a variety of classification and diagnosis methods. However, when the severity of the disease is different, there is not much difference between the DR images, and the feature extraction and classification work are difficult to perform well [19].

As a multidomain interdisciplinary subject, machine learning has been greatly developed in recent years. Deep learning can be used to mine deep features of data due to its powerful feature extraction capabilities. At present, many scholars use machine learning algorithms to study the data of diabetic patients to improve the treatment effect and condition of diabetic patients. Generally speaking, these research methods can be divided into mathematical statistics methods and machine learning methods. However, in order to achieve the purpose of using diabetes data mining to realize the purpose of auxiliary diagnosis and treatment with practical value, more in-depth research is needed.

Computer is used to classify the image, the pixel points of the image are converted into features, the neural network is used to analyze the characteristics of the image, and the target image is classified according to the feature information. The use of computer technology can perform automatic diagnostic analysis and rapid processing of fundus images, which can greatly reduce the workload of professional ophthalmologists. Doctor can not only obtain the classification result according to the model, but also can remove the influence of the photograph of the environment through the preprocessing method and obtain a clearer fundus image. The doctor can further improve the accuracy of the diagnosis by combining the results given by the computer. Image classification is a hot topic recently. It is meaningful to study the use of intelligent methods to automatically analyze medical images to assist doctors in achieving efficient diagnosis of diseases [20].

All in all, with the continuous development of image processing, convolutional neural network, and other technologies, medical image processing has shown broad development prospects and plays an important role in the rapid and accurate diagnosis and treatment of certain diseases. DR data processing by computer, combined with traditional image processing and deep learning methods to screen and diagnose data, can greatly improve the efficiency and accuracy of DR diagnosis, which is of great significance to doctors and patients. Using this method can adjust the treatment plan for the patient in time; it is a subject worth studying, and the research on this subject has certain practical significance and scientific research value.

## 2. Convolutional Neural Network

With the continuous deepening of the network structure, its ability to express features is gradually strengthened. The deep convolutional neural network model, which is based on the traditional neuron model, has been widely used in the field of image processing. Convolutional neural networks reduce the number of parameters by using local receptive fields for weight sharing. Each neuron only perceives the data of this layer, and the higher perception layer combines the underlying data to obtain global data, greatly reducing the number of parameters. This part mainly introduces the convolutional neural network and the classic convolutional neural network model in image classification. A neural network is formed by connecting neurons one by one. The difference between a convolutional neural network and a traditional neural network is that the convolutional neural network contains a feature extractor composed of convolutional layers and subsampling layers. As shown in Figure 1, a convolutional neural network consists of an input layer, a convolutional layer, a fully connected layer, and an output layer.

### 2.1. Convolutional Layer

In convolutional neural networks, the process of feature extraction is carried out in convolutional layers. The features extracted by low-level convolution and high-level convolution are different. Low-level features such as edges, lines, corners, and textures are usually extracted by low-level convolution layers. Complex information of images is often extracted by high-level convolution layers, which is obtained by layer extraction, so as to complete the extraction of the global information of the image. The image is passed to the convolution kernel through the input layer to perform the convolution operation, and then the excitation function is used to process the result of the convolution operation to obtain the feature map. The calculation formula of the convolutional layer is:

(1) $$\begin{array}{c} y_{n}^{l}=f_{l}\left(\underset{m\in V_{n}^{l}}{\sum }y_{m}^{l-1}w_{m,n}^{l}+b_{n}^{l}\right). \end{array}$$

Among them, *y* is the *n*th feature map in the *l*th layer of the convolutional neural network, *f* represents the activation function, *b* is the bias term, and *V* is the input feature map set.

Activation function is used to increase the nonlinear factor of the convolutional neural network. The widely used activation functions are the sigmoid function, tanh function, and ReLU function. The expression for the sigmoid function is

(2) $$\begin{array}{c} f\left(z\right)=\frac{1}{1+e^{-z}}. \end{array}$$

It can be known from the sigmoid function that its value is between (0, 1), and the output can be mapped to between (0, 1), which is shown in Figure 2. It is usually used in binary classification problems. The disadvantage of this function is that the derivation is complex, and the amount of calculation is large when backpropagation is performed. And the derivatives at both ends of the function are close to 0, which will cause the gradient to disappear in the backpropagation of the deep network.

The expression of the tanh function is

(3) $$\begin{array}{c} f\left(z\right)=\tanh\left(z\right)=\frac{e^{z}-e^{-z}}{e^{z}+e^{-z}}, \end{array}$$

(4) $$\begin{array}{c} \tanh\left(z\right)=2sigmoid\left(2z\right)-1. \end{array}$$

It can be known from the tanh function that the value range of the tanh function is between (-1, 1), which is shown in Figure 2. Compared to sigmoid, the output of the tanh function is centered at 0 and has a wider output range. However, after the derivation of both ends of the same function, it is close to 0. It is easy to cause the gradient to disappear, which is not conducive to the training of deep network.

The expression of the ReLU function is

(5) $$\begin{array}{c} f\left(z\right)=\max\left(0,z\right). \end{array}$$

### 2.2. Pooling Layer

Pooling layers are also known as downsampling layers. Adding a pooling layer after the convolution operation can effectively reduce the parameters and avoid the computer computing pressure caused by the large amount of parameter data. This reduces the amount of data processing while retaining useful information and also speeds up the training of the network. Generally, pooling is divided into max pooling and average pooling. Maximum pooling is generally used when reducing dimensions and can extract the main features, while average pooling averages the features and does not contribute to the extraction of the main features. The feature calculation formula of the pooling layer is as follows:

(6) $$\begin{array}{c} y_{n}^{l}=f_{l}\left(z_{n}^{l-1}w_{n}^{l}+b_{n}^{l}\right). \end{array}$$

### 2.3. Fully Connected Layer

In the convolutional neural network, the role of “classifier” is usually played by the fully connected layer, which can be classified according to the combination of features. It usually exists in the later layers of the convolutional neural network. The feature position brings the accuracy of classification. The adverse effects can be effectively reduced by the fully connected layer. It can be regarded as a conventional artificial neural network introduced in the previous section and works in the same way as the artificial neural network. The output formula of the fully connected layer neuron is shown below.

(7) $$\begin{array}{c} y_{n}^{l}=f_{l}\left(\overset{N_{l}-1}{\underset{m=1}{\sum }}y_{m}^{l-1}w_{m,n}^{l}+b_{n}^{l}\right). \end{array}$$

### 2.4. Training of Convolutional Neural Networks

Convolutional neural networks often use the backpropagation method to learn and optimize parameters. The loss function is used to judge the gap between the actual value and the predicted value, and different optimizers are selected to update and calculate the network parameters of the model to make it approximate or reach the optimum value.

The loss function is used to represent the error between the actual calculation result and the expected output result. The smaller the loss function, the better the model learning data. Often, the distance between the predicted value and the true value can be estimated simply by using the mean squared error (MSE), which is given by

(8) $$\begin{array}{c} MSE=\frac{\sum_{i=1}^{n}{\left(y_{i}-{\overset{\wedge }{y}}_{i}\right)}^{2}}{n}. \end{array}$$

Taking a single sample as an example, *z* is the real value, *b* is the activation value *∂*(*z*), and *z* is the neural network output *wx* + *b*. The mean square error loss function can be written as

(9) $$\begin{array}{c} MSE=C=\frac{{\left(y-a\right)}^{2}}{2}. \end{array}$$

In the training of the convolutional neural network, the weight parameters are updated by taking the partial derivatives of *w* and *b*, and the results are

(10) $$\begin{array}{c} \frac{\partial C}{\partial \omega }=a\sigma^{\prime }\left(z\right), \end{array}$$

(11) $$\begin{array}{c} \frac{\partial C}{\partial b}=a\sigma^{\prime }\left(z\right). \end{array}$$

If it is a convolutional layer, for each convolution kernel, the weights and biases are updated as follows:

(12) $$\begin{array}{c} W^{l}=W^{l}-\alpha \overset{m}{\underset{i-1}{\sum }}\delta^{i,l}a^{i,l-1}, \end{array}$$

(13) $$\begin{array}{c} b^{l}=b^{l}-\alpha \overset{m}{\underset{i-1}{\sum }}\underset{\mu ,\upsilon }{\sum }\delta^{i,l}. \end{array}$$

## 3. Diabetes Data Analysis and Processing

The experimental data for this research topic were case data from 10 years of admission records of diabetic patients in 130 hospitals across the United States. Due to the huge amount of data in this dataset, the first thing to do in this research for such a dataset is to perform basic analysis and data screening on the dataset to gain a preliminary understanding of the content of the dataset. The dataset has a total of 10766 samples, 49 attribute columns, and 2 label variables. The label variable 0 means the patient was not readmitted within 30 days of discharge, and 1 means the patient was readmitted within 30 days. The label of the patient's admission record is used to judge whether the patient is likely to be readmitted in a short period of time, so as to judge the effect of this treatment. Among them, each sample includes 49 attributes, such as patient number, race, gender, and age. This study divides these attributes into four dimensions: (1) the patient's basic physiological information, including weight, race, and gender; (2) the patient's basic admission registration information, including the patient's admission number and admission time; (3) the patient's condition diagnosis records; and (4) records of patients' medication information. This paper uses machine learning algorithms to mine the hospitalization records of diabetic patients. Then this paper explores the potential treatment experience and predicts the development of the patient's condition, so as to improve the treatment efficiency and treatment effect of the patient.

With reference to the opinions of hospital physicians, this study firstly performed manual classification of the features in the dataset. In this dataset, the age, gender, weight, and other information of patients have been fully confirmed to have an impact on diabetes. Through observation of the dataset, it is found that the patients admitted to the hospital include different races. Considering that race may be a potential factor for the onset of diabetes, so add it to the data dimension. Secondly, this study selected biochemical indicators related to diabetes, which mainly include fasting blood glucose value, glycosylated hemoglobin value, and insulin release test. Among them, the blood sugar level can be reflected and is an important criterion for judging the changes in the condition of diabetic patients. Glycated hemoglobin is formed by the combination of hemoglobin in red blood cells and sugars in serum, and its content depends on the blood glucose concentration and the contact time between blood glucose and hemoglobin. Therefore, it can be used as an important indicator for diabetes monitoring; the insulin release experiment can reflect whether the function of the insulin-secreting *β* cells in the patient's pancreatic islets is normal. These biochemical indicators can provide important reference for doctors to diagnose the disease and also have important value for the experimental purpose of this study. In attribute selection, this study also selected doctors' diagnostic records and medication records as key attributes.

Since the dataset used in this experiment is the original dataset recorded by the hospital, there are problems such as inconsistent data format, incomplete data, and data recording errors in the dataset. Since the quality of the data determines the upper limit of the analytical performance of the model, this section focuses on data cleaning.

An important task of data cleaning is to deal with missing values in the original dataset. The main reasons for the lack of data in the medical records are that the medical staff misses the records or does not obtain a certain record of the patient. Generally, there are three main methods for dealing with missing values: delete records, data imputation, and no processing.

If only a small number of records can be deleted to achieve the set goal, the method of deleting missing values is effective, but this method has great limitations, wastes a lot of data resources, and discards a large number of records hidden in these records. The methods of data interpolation mainly include the use of fixed values for interpolation; the use of known points to establish appropriate interpolation functions for interpolation; and the use of mean/median for interpolation. Since some models can treat missing values as a special value and allow modeling on missing values, missing values are not handled.

## 4. Simulation Analysis

A total of 307 epochs were trained in the experiment, and the learning rate change curve during the whole training process is shown in Figure 3. The accuracy and loss curves for training and validation sets are shown in Figure 4. By comparing the quasi-curvature curve and the loss curve, it can be found that the simulation has 200-300 epochs after training, the accuracy on the training set and the accuracy on the validation set gradually become stable, and the accuracy on the training set after 250 epochs is stable. The rate is basically stable, and the accuracy rate on the validation set also oscillates within the stable range. At the same time, during the whole training process, the training loss curve kept a steady decline, and the validation set loss curve oscillated and decreased. After 200 epochs, the oscillation amplitude became larger, and after approaching 300 epochs, the oscillation amplitude increased especially obviously, and there was a certain increase in trend. In summary, it can be considered that the model gradually stabilizes in fitting ability after epoch is 200. For this reason, in this experiment, the model with epoch in the range of 200-305, which performed well in the accuracy and loss rate of the validation set, was tested on the final 53575 test set.

Experiment 2 trains a total of 445 epochs, and the learning rate changes during the training process, as shown in Figure 5. By comparing the quasi-curvature curve and the loss curve, it can be found that after the simulation has 350-450 epochs after training, the accuracy on the training set and the accuracy on the validation set gradually become stable, and the accuracy on the training set after 400 epochs is basically stable, and the accuracy rate on the validation set also oscillates in the stable range. At the same time, during the whole training process, the training loss curve keeps decreasing steadily, and the validation set loss curve oscillates and decreases. At about 350 epochs, the oscillation amplitude still stays stable.

In summary, it can be concluded that the model gradually stabilizes in fitting ability when epoch is bigger than 350. For this reason, the epoch around 350-450 was selected for this experiment, and the model has good accuracy and loss rate in the validation set. The obtained specificity, sensitivity, and accuracy rate turns out that it is the best model.

In this paper, a data preprocessing method based on CNN is proposed, which is compared with the traditional normalization preprocessing method. After Gaussian filtering, it is fused with the original image to eliminate noise information, and the gamma correction method is used to eliminate the influence of high exposure and underexposure. The experimental chart is shown in Figure 6. It can be seen from the figure that the data of the preprocessing methods gradually increases with the training accuracy of the 0~20 generation model and then tends to be flat, and the results fluctuate around the final value. At the beginning, because the network model is preprocessed, the accuracy of the model changes greatly when verifying the preprocessing method proposed in this paper, the graph shows an upward trend, the slope is large, and the accuracy increases rapidly. Compared with the original method, the accuracy rate of the method is small, but the final accuracy rate is higher than the original single method. That is, the accuracy rate is increased by 0.7% compared with the previous method. The results show that the various preprocessing methods proposed in this paper can improve the classification accuracy.

In addition, in order to further verify the effectiveness of the proposed model, the images were processed by traditional matched filtering, morphological methods, proposed improved matching filtering, and morphological fusion scheme. The result is also compared with the expert manual segmentation results. For the retinal blood vessel segmentation of the fundus, the retinal blood vessel segmentation method given in this paper has a certain improvement in effect compared with the morphological method and the matched filtering method, and the accuracy and sensitivity are improved, and specificity, the retinal vessel segmentation method in this paper performs better, and its value is also improved. In order to intuitively compare the effects of various methods on blood vessel segmentation in retinal images, three retinal images were selected from two publicly available DRIVE and STARE datasets, which are commonly used in retinal blood vessel segmentation, and processed with three methods, respectively. The algorithm proposed in this paper has a good segmentation effect, can segment most of the tiny blood vessels, and can restore the blood vessel feature information better. This is because the Hessian matrix is used to obtain the direction of the blood vessels in the retinal blood vessel segmentation scheme given in this paper, so as to guide the filtering angle of the matched filter, so the accuracy of the segmentation is improved, and the multiscale operation can better improve the blood vessel details, so that most of the tiny blood vessels can be segmented.

### 4.1. No Data Balance Predicts Short-Term Readmission Risk for Diabetes

In order to verify the effectiveness of hospital case data balancing, this study tested the classification prediction method proposed in this study by observing the experimental results and using the data without data balancing processing. The experimental results are shown in Figure 7. The experimental classification model with the dataset and no data balance has a prediction accuracy of 0.81, a recall of 0.84, a specificity of 0.73, and a precision of 0.71.

### 4.2. Predicting Short-Term Readmission Risk in Diabetes by Data Balancing Processing Datasets

In order to verify the necessity of data balance, this study conducted training on the data after data balance. In this study, CNN was used to predict color patches of 6∗6 pixels, with a total of 180,818 pieces of data.  Figure 8 shows that the classification accuracy of the CNN model is 0.837. It can be seen that the model predicts the trend of diabetes more accurately, and the variance value of the algorithm is small, indicating that the algorithm has good stability. The recall of the algorithm was 0.902, the accuracy of the model was 0.741, and the specificity of the model was 0.79. Combining these indicators, it can be seen that the performance of the model is good and the recall rate is high. The results showed that the model had a lower probability of misjudging patients with poor recovery as good recovery, and the prediction was more accurate.

## 5. Conclusion

In this paper, a convolutional neural network is used to establish a diabetes prediction model. In the model, there are mainly four parts: data collection, data analysis and processing, initial feature selection, classification prediction, and algorithm validity test. The conclusions are drawn as follows:

1. First of all, the dataset can be used as a representative of the diabetes dataset. It is not only rich in features, but also has a large number of experimental samples, which has the characteristics of good representativeness
2. Combined with the opinions of the doctors in the hospital, the dataset was classified and analyzed filled with data. The abnormal data was detected, and the features were sorted by contribution degree. The features that are irrelevant to the experimental purpose were eliminated after combining with the doctor's opinion, and the data features were preliminarily processed
3. The processed data is fed into a CNN model for training, and classification results are obtained. However, since the research purpose of this study is to assist physicians in the diagnosis and treatment of diabetic patients in areas with limited medical resources, the prediction results of this model are still in the research stage, and there is still a certain distance from practical application

## Figures and Tables

**Figure 1:** Convolutional neural network.

**Figure 2:** Figures of the functions.

**Figure 3:** Learning rate change curve in experiment 1.

**Figure 4:** Accuracy and loss rate curves.

**Figure 5:** Learning rate change curve in experiment 2.

**Figure 6:** The comparison with different preprocessing methods.

**Figure 7:** Prediction of short-term readmission risk of diabetes mellitus without data balancing.

**Figure 8:** Predicting short-term readmission risk in diabetes by data balancing processing datasets.

## Data Availability

The experimental data used to support the findings of this study are available from the corresponding author upon request.
